RETRACTED

# Staged Surgical Management in the Treatment of Primary Epidural Hydatidosis of the Spine: A Case Series and Review

**DOI:** 10.7759/cureus.401

**Published:** 2015-12-12

**Authors:** Ameya S Kamat, Crispin Thompson, Mohammed Ben Husien

**Affiliations:** 1 Department of Neurosurgery, Groote Schuur Hospital, University of Cape Town

**Keywords:** spinal hydatidosis, staged management

## Abstract

Hydatid disease is a parasitic infection linked to the Echinococcus granulosus tapeworm. Infected cysts can present anywhere in the human body, but the liver is the most frequently involved organ, followed by the lungs. The prognosis is generally poor and may be comparable to that of neoplastic disease. Primary spinal hydatidosis accounts for less than 1% of all cases and virtually all these cases have extradural involvement. We describe a case review consisting of two patients who presented over a three week period with primary spinal extradural hydatidosis in the Western Cape region of South Africa. Both patients presented with lower limb paraparesis and were treated aggressively with two-stage surgical procedures, resulting in a dramatic improvement in their neurological status.

## Introduction

Hydatid disease is a parasitic infection linked to the Echinococcus granulosus tapeworm. Infected cysts can present anywhere in the human body, but the liver is the most frequently involved organ, followed by the lungs. Hematogenous dissemination may arise in almost any anatomic location, including the spine [1]. The first description of spinal hydatid disease was made by Churrier in 1807. Despite the introduction of advanced surgical and pharmacological therapy, the management of spinal hydatid disease continues to be a challenge and the disease is prone to recurrence. The cystic infestation aggressively invades the spinal column, leading to its eventual destruction, and resulting in neurological compromise. The prognosis is generally poor and may be comparable to that of neoplastic disease [2]. Primary spinal hydatidosis accounts for less than 1% of all cases and virtually all these cases have extradural involvement [2]. Isolated primary spinal intradural hydatidosis is a very rare condition, occurring in less than 0.1% of spinal hydatid cases and, hence, only a few cases have been previously documented [3-5].

We describe a case review consisting of two patients who presented over a three week period with primary spinal extradural hydatidosis in the Western Cape region of South Africa. Both patients presented with lower limb paraparesis and were treated aggressively with two-stage surgical procedures, resulting in a dramatic improvement in their neurological status. Appropriate written consent was obtained from the relevant parties.

RETRACTED

## Case presentation

### Case 1

A 41-year-old male presented with a three-week history of progressive limb weakness resulting in loss of mobility. Significant past history included thoracic laminectomy for evacuation of spinal hydatid cysts 6 and 11 years previously, after which the patient made a good neurological recovery, and a right-sided thoracotomy for excision of intrathoracic hydatid cysts. Pertinent clinical findings included power in 3/5 of all muscle groups in both lower limbs and mildly increased tone. The patient was not able to mobilize. Bladder and bowel function was intact. Magnetic resonance imaging (MRI) of the thoracic spine demonstrated an extradural, non-enhancing, multiloculated, polycystic lesion with involvement of the T8 vertebral body. The lesion exhibited low signal intensity on T1-weighted and high signal intensity on T2-weighted sequences (Figure 1).

**Figure 1:** Axial T2-weighted MRI of the thoracic spine demonstrating invasive hydatidosis

The spinal cord was compressed and displaced anterolaterally. The lesion was entirely extradural (Figure 2).

**Figure 2:** Coronal T2-weighted MRI of the thoracic spine demonstrating invasive hydatidosis

Chest radiograph showed dystrophic calcification over the inner curvature of the right posterolateral ribs. Abdominal ultrasonography was essentially normal. There was no evidence of current hepatic or pulmonary hydatid disease. The patient underwent a two-stage procedure. Firstly, a revision laminectomy was performed for removal of the extradural cysts within the spinal canal, along with a bilateral T8 transpedicular excision of the posterior component of the T8 vertebral body, for decompression of the spinal cord. This necessitated the removal and replacement of previously placed titanium rods. This was followed by a transthoracic T8 vertebrectomy with the insertion of a humeral shaft allograft strut (Figure 3).

**Figure 3:** Lateral plain film radiograph post-fusion and strut allograft insertion of thoracic spine

Intraoperative findings confirmed a multitude of white cystic extradural lesions of various sizes displacing and compressing the thoracic spinal cord. The cyst fluid was macroscopically clear. The surgical site was irrigated thoroughly with warm hypertonic saline to aid in the eradication of liberated scolices and reduce the risk of recurrence. Postoperatively, the patient made a good neurological recovery and was able to mobilize unassisted. During the perioperative period, the patient was covered with albendazole and praziquantel, and he was subsequently discharged on life-long albendazole therapy.

RETRACTED

### Case 2

A 19-year-old female with known previous spinal hydatid disease presented with progressive lower limb weakness over a three month period, resulting in profound paraparesis. The patient had undergone several previous hydatid cyst evacuation procedures. She had normal bladder and bowel function. Examination findings revealed severely decreased power (2/5) in all lower limb muscle groups with mildly increased tone. Perianal sensation and anal tone were preserved. MRI of the spine demonstrated an extradural, multi-loculated, non-enhancing lesion involving the T8 vertebra with extension into the thoracic spinal canal, resulting in compression of the spinal cord (Figure 4). The disease was also present in the prevertebral region with extension into the mediastinum. The lesion exhibited low signal intensity on T1-weighted and high signal intensity on T2-weighted sequences. Computerized tomography (CT) of the abdomen demonstrated a hypoechogenic mass in the liver consistent with a hemangioma. Plain film chest radiographs were unremarkable. The patient underwent a two-stage procedure. Firstly, a T7-T9 posterior decompression and instrumented fusion were performed. The second procedure involved a transthoracic anterior vertebrectomy and insertion of a humeral shaft allograft strut.

**Figure 4:** Axial T2-Weighted MRI demonstrating spinal cord compression

Intraoperative findings showed a multicystic lesion displacing and compressing the thoracic spinal cord. The cyst fluid was macroscopically clear. The surgical site was irrigated thoroughly with warm hypertonic saline to aid in the eradication of liberated scolices and reduce the risk of recurrence. Postoperatively, the patient made a good neurological recovery and was discharged home being able to mobilize unassisted. She was treated with life-long albendazole therapy.

## Discussion

Despite hydatidosis being rare in westernized nations, cases have been reported in Western Europe, the United States of America, New Zealand, and Australia. It is much more common in endemic areas, however, such as certain Mediterranean regions, Eastern Europe, East Africa, and parts of South Africa [6-7]. Unlike hepatic and pulmonary disease, central nervous system involvement occurs in only 0.5-1% of patients [2-5, 8].

Echinococcus granulosus has definitive and intermediate hosts, as do other cestodes. The adult worm lives in the jejunum of the definitive host, usually the domestic dog or other carnivores. The parasite has a gravid proglottid that is shed in the faeces of the dog and subsequently ruptures, thereby releasing hundreds of ova that are incidentally ingested by sheep, cows, or humans (intermediate hosts). In the intermediate hosts, after digestion, the outer layer embryos (oncospheres) develop in the small bowel to penetrate the duodenal mucosa and disseminate via the portal circulation, following which they either develop into cysts or are destroyed by the hosts’ immune response [9-12].

RETRACTED

The liver is the most commonly involved site, followed by the lungs. Primary spinal hydatidosis accounts for less than 1% of all cases with the majority having extradural involvement [2, 13-15]. However, isolated primary spinal intradural hydatidosis is a very rare condition, occurring in less than 0.1% of spinal hydatid cases, and hence, only a few cases have been previously documented [3-6].

Bone involvement, albeit rare, has been reported and in many cases that involve the spine. Disease infestation is thought to begin in the center of the vertebral body and may extend into the spinal canal or paravertebrally, involving the erector spinae muscles, costal muscles, or paravertebral soft tissues [3]. Intradural extramedullary involvement is found in 9% of the cases [8-10].

Primary infestation of the spine is thought to occur through the portovertebral shunts involving the center of the vertebral body [11]. Penetration by larvae of the vertebral cancellous bone causes diffuse cortical weakening due to compression or avascular necrosis [16-17]. This can lead to pathological fractures of the vertebral body, laminae, and pedicles. If the cysts die, dystrophic calcification occurs, which can be seen on plain film radiographs. Eventually, the infestation may extend beyond the vertebral body with the formation of a space-occupying lesion, resulting in symptoms of spinal cord or nerve root compression [18].

The clinical symptomology of the spinal disease usually occurs several years after the initial infestation of cysts. This is because cysts grow slowly over several years and are most likely limited by the resistance of the surrounding bone. Most patients report a prolonged history of back pain that may be accompanied by radicular symptoms [19]. Cyst rupture, both preoperatively and intraoperatively, can be associated with spillage of the scolices. This may result in a spectrum of hypersensitivity reactions from pruritus, urticaria, and edema to anaphylactic shock [20]. Thus, the preoperative diagnosis of hydatid disease is of great importance.

A diagnosis of hydatid disease should be considered in cases of spinal cord compression in endemic countries. Detection of antibodies for echinococcal polypeptide antigens has a high degree of specificity. ELISA has a high sensitivity and specificity in abdominal disease, but is low in extra-abdominal disease [17]. From a radiological perspective, spinal CT scans show good bony resolution and demonstrate erosions within cancellous bone in the absence of periosteal reaction. MRI, however, is the radiological modality of choice as it has superior soft tissue resolution. The lesion has a bunch-of-grapes appearance or multiple cystic cavities. The signal characteristics of the cyst content on MRI is similar to CSF [18]. On T1-weighted images, the cyst wall appears only slightly more hypointense than the cyst content and enhances very slightly post-administration of gadolinium.

RETRACTED

Surgical management is currently considered the treatment modality of choice for spinal hydatid disease [7, 15, 21]. Anterior or posterior approaches may be considered. Many surgeons utilize a two-stage procedure incorporating both anterior and posterior approaches. This is the method of choice at our institution. Vertebral involvement is a major challenge for surgeons. As the lesion is highly infiltrative, spillage of scolices is often unavoidable during surgery. Historically, it seems that simple decompression by means of a laminectomy was by far the most commonly utilized procedure [19-20]. This approach allows simple and straightforward decompression with few complications. The major limitation of a laminectomy, however, is that access to the vertebral body is limited. This raises concerns as the vertebral body is often affected in spinal hydatidosis. Due to these limitations, the risk of disease progression and recurrence is high with laminectomy alone. Extensive bony resection with stabilization and grafting has been shown to prolong survival due to decreased recurrence and slower progression rates [20-21]. A few centers have advocated using two-stage procedures. This includes initially utilizing a posterior approach to perform a laminectomy and instrumented fusion. The next stage utilizes the anterior approach. Anterior corpectomy or vertebrectomy with the insertion of an allograft strut may be performed. This approach proved to have the lowest recurrence rate and has been used by our spinal surgical team with good results [21].

Pharmacological intervention has a role in spinal hydatidosis. Drug therapy with albendazole is the recommended agent. Although this drug does not cure spinal hydatid disease, it does slow progression and decreases recurrence rates and ought to be used in conjunction with surgery [2]. It has been reported that praziquantel is also effective against Echinococci, either alone or in combination with albendazole [3, 20]. Current treatment protocols at our institution recommend a combined therapy during the perioperative period, followed by life-long albendazole monotherapy.

RETRACTED

## Conclusions

Spinal hydatid disease, especially in endemic areas, must be considered in the differential diagnosis in patients with spinal cord compression, back pain, or radicular symptoms. Primary epidural hydatid disease is a rare condition. Surgical decompression is the treatment of choice using either a posterior approach or a combined posterior and anterior approach. As the disease is highly invasive, surgery is rarely curative; however, the recurrence rates and the time between recurrences are improved using more aggressive surgical approaches to treatment. This entails extensive bony resection using a posterior and anterior approach. The advantage of using instrumentation is that it aids in vertebral stability. Our case review and operative experience shows that the outcomes are improved with this strategy. Adjuvant drug therapy during the perioperative period and intraoperative lavage with hypertonic saline may further reduce the incidence of recurrence. Despite even the most extensive resections, the disease has a high propensity for recurrence that may eventually lead to progressive destruction of the vertebral column and subsequent neurological compromise. 
